# Clinical Effect of Arthroscopic Resection of Extra-Articular Knee Osteochondroma

This article has been retracted.

**DOI:** 10.3390/jcm12010052

**Published:** 2022-12-21

**Authors:** Peng Chen, Li Shen, Qiong Long, Wei Dai, Xiaocheng Jiang, Canfeng Li, Jianwei Zuo, Jiang Guo, Xintao Zhang

**Affiliations:** 1 Department of Sports Medicine, Peking University Shenzhen Hospital, Shenzhen 518036, China; 2 Shenzhen Healthcare Committee Office, Shenzhen 518020, China

**Keywords:** arthroscopy, extra-articular knee, osteochondroma

## Abstract

**Objective**: The aim of this study was to investigate clinical outcomes of arthroscopic resection of extraarticular knee osteochondroma. **Methods**: A retrospective analysis was performed in 74 patients with extra-articular knee osteochondroma treated by arthroscopic resection between August 2011 and August 2021, including 43 males and 31 females. Overall, 26 Distal femur cases and 48 proximal tibia cases were involved, with an average age of 31.7 ± 11.3 (11–57) years. Preoperative routine knee X-ray, CT, and MRI were performed before the operation. The Lysholm knee score, International Knee Documentation Committee (IKDC) score, Tegner knee motor function score, and visual analogue scale (VAS) were used to evaluate symptoms and functions before surgery and 3, 6, 12, and ≥24 months after surgery. **Results**: The average course of disease was (7.9 ± 3.7) months (range, 3–14 months) in 74 patients. The average follow-up was (22.6 ± 6.4) months (range, 10–37 months). There were no cases of vascular or nerve injury or wound infection. Compared with the preoperative function, the average scores of VAS, Lysholm, IKDC, and Tegner joint motor function decreased or increased significantly compared with the last follow-up (3.6 ± 1.1 vs. 0.1 ± 0.02, 44.5 ± 2.3 vs. 91.3 ± 4.9, 53.7 ± 2.6 vs. 94.2 ± 5.1, 4.6 ± 1.2 vs. 9.4 ± 1.4, *p* < 0.001). There was no recurrence or metastasis during the follow up. **Conclusions**: With the advantages of less trauma, high precision, less pain, and rapid recovery, arthroscopic resection of extra-articular knee osteochondroma can significantly improve the function of knee. It can be gradually extended to the treatment of other benign bone tumors.

## 1. Introduction

Osteochondroma is the most common benign bone tumor, occurring mostly in the distal femur and proximal tibia [1]. Although the malignant transformation rate of osteochondroma is only 1–2% [2], patients still need operation treatment because of the symptoms of tumor compression on adjacent tendons, nerves, muscles, or blood vessels. For extra-articular osteochondroma, open surgical resection is still the conventional treatment method [3,4,5], but this technique increases the risk of infection and may lead to joint stiffness, dysfunction, and other issues, with complication rates ranging from 11.7% to 12.5% [3,4], including arterial tears, compartment syndrome, fractures, and nerve palsy.

Arthroscopic surgery has become the preferred treatment method for patients who have joint diseases because of its reduced trauma and good curative effect [6,7]. In recent years, with the development of arthroscopic equipment, technique, and the gradual popularization of the minimally invasive concept, the arthroscopic technique has become more and more widely used outside the joints [8,9,10]. This enables minimally invasive resection of benign bone tumors, resulting in smaller surgical incisions, more complete tumor resection, and fewer postoperative complications. This article retrospectively analyzes 74 patients with extra-articular osteochondroma of the knee treated by arthroscopy in our department from August 2011 to August 2021. We hope this study can provide a reference for the application of endoscopy in other benign bone tumors.

## 2. Materials and Methods

### 2.1. Inclusion and Exclusion Criteria

Inclusion criteria: The patient expressed his consent to arthroscopic surgery. All examinations showed that the tumor had clear borders and no obvious adhesion to surrounding tissues. The tumor was located in the distal femur or proximal tibia, and it could be basically diagnosed with osteochondroma. Biopsy pathology was performed before surgery if the nature of the tumor could not be determined.

Exclusion criteria: The demarcation between the tumor and surrounding tissues was unclear. The tumor could not be determined to be benign before surgery. There were major blood vessels or nerves around the tumor. The patient disagreed with this surgical plan. 

### 2.2. Patient Selection

This study is a retrospective research, which was approved by institutional review board of our hospital (2017009). All patients underwent X-ray and CT preoperatively, and MRI was performed if needed (Figure 1A,B). Among the 74 patients, 43 were male, and 31 were female. The average age was 31.7 ± 11.3 years (11–57 years), and all patients complained of local mass and tenderness. X-ray showed a single osteochondroma, with 26 cases of distal femur and 48 cases of proximal tibia. The tumor size of the patients ranged from the smallest, 1 × 1 × 1 cm^3^, to the largest, 2 × 2 × 3 cm^3^. The postoperative pathological examination of all the 74 cases confirmed osteochondroma. The average follow-up period was 22.6 months (10–37 months). 

### 2.3. Surgical Technique

The surgical procedures were performed with the patient in a supine position under general anesthesia; the tumor border and its surrounding important blood vessels and nerves were marked on the body surface preoperatively with the help of ultrasound; and a pneumatic tourniquet was placed on the root of the thigh.

Two arthroscopic incisions were made at the upper and lower side of the tumor mark, followed by local blunt dissection with vascular forceps or periosteal exfoliator, reaching the bone surface and creating a cavity. After the arthroscope was placed, the local soft tissue was cleaned with a shaver to expose the tumor tissue and its borders (Figure 1C), and part of the tumor tissue was removed with a nucleus pulposus forceps and sent for rapid pathological examination during the operation (Figure 1D). After the benign tumor was confirmed, arthroscopic resection was performed. First, the cartilage cap was burned off with a radiofrequency knife, and then, the tumor was completely removed from the root of the tumor with an osteotome. If the tumor was too large, it could be cut into small pieces with a nucleus pulposus forceps and then taken out (Figure 1E,F). In order to avoid tumor tissue’s dissemination and colonization into other parts or causing the surgical site to excessively swell, attention was paid to maintaining smooth drainage of the irrigation fluid during the operation. There was no need to place drainage after surgery, but an elastic bandage was used for local compression. As soon as the wound pain was relieved postoperatively, passive flexion and extension of the knee and weight-bearing activities were conducted, and the X-ray inspection was reviewed (Figure 1G). The final diagnosis depended on the postoperative pathological results (Figure 1H).

### 2.4. Clinical Assessment

Limb function evaluation indicators include Lysholm score, International Knee Documentation Committee (IKDC) score, Tegner knee motor function score, and visual analog scale (VAS) pain score. Knee function and pain were assessed before surgery at 3, 6, 12, and ≥24 months after surgery. X-ray was reviewed at the first day and each assessment point postoperatively to confirm if the tumor had recurred.

### 2.5. Statistical Methods

All data were statistically analyzed with SPSS 25.0 (IBM, Armonk, NY, USA), and the function data were expressed as “mean ± standard deviation”. Paired *t*-test was used for continuous variables. *p* < 0.05 was considered statistically significant.

## 3. Results

Among the 74 patients, the duration from symptom onset to surgery was 7.9 ± 3.7 months (3–14 months). The postoperative follow-up was 22.6 ± 6.4 months (10–37 months). The pain of the patients was significantly relieved after the operation, and the VAS score decreased from 3.6 ± 1.1 points preoperatively to 0.1 ± 0.02 points at the last follow-up (*p* < 0.001) (Table 1).

The Lysholm score increased from 44.5 ± 2.3 points preoperatively to 91.3 ± 4.9 points at the last follow-up (*p* < 0.001); the IKDC score increased from 53.7 ± 2.6 points preoperatively to 94.2 ± 5.1 points (*p* < 0.001); the Tegner score increased from 4.6 ± 1.2 points preoperatively to 9.4 ± 1.4 points (*p* < 0.001) (Table 1). During the follow up, there were no complications such as wound infection, poor wound healing, bleeding, fracture, prolonged swelling, neurovascular injury, surrounding tendon injury, deep vein thrombosis, or local hematoma in all patients. Three patients had mild local tenderness 6 months after operation, and their symptoms were relieved after symptomatic drug treatment and physical therapy. There was no tumor recurrence in this group of patients during the follow-up period.

## 4. Discussion

Extra-articular osteochondroma of the knee presents as a single or multiple event in childhood and adolescence [11,12], and intra-articular osteochondromas are very rare [13]. Genetic studies [14,15] show that hereditary osteochondromas are associated with exoskeleton protein-1 (chromosome 8q24.1), -2 (chromosome 11p13), and -3 (chromosome 19 in the short arm) sites. Both extra-articular and intra-articular osteochondromas can cause pain, discomfort, and joint mobility limitation.

The only effective treatment for osteochondromas is surgical excision. For intra-articular osteochondroma, most orthopedic surgeons have accepted the surgical method of arthroscopic resection, and the effect has also been generally recognized. Ayerza et al. [16] reported that seven cases of intra-articular osteochondroma of the distal femur were resected under arthroscopic surgery. After an average follow-up of 33 months, the pain symptoms of the patients were significantly relieved, the function of the joint also returned to normal, and there were no postoperative complications. Many other surgeons [17,18,19,20,21] have also tried this procedure and performed arthroscopic resection of intra-articular osteochondroma, and all achieved good surgical results without postoperative complications.

However, the application of arthroscopy in extra-articular osteochondromas is still in the exploration stage. Aalderink et al. [22] reported a case of arthroscopic resection of osteochondroma of the scapula. The patient was placed in the prone position, and the tumor was completely removed with a rongeur. After the resection, the patient returned to normal activities 6 weeks after surgery. Fukunaga et al. [23], Perez et al. [24], and van Riet [25] used similar surgical procedures to excise osteochondroma of the scapula. All patients recovered well after surgery, with no postoperative complications and no tumor recurrence during follow-up. In addition, Gudas et al. [26] also used arthroscopic technique to successfully resect the fibular capitulum osteochondroma without injury to the common peroneal nerve. Khosla et al. [27] reported arthroscopic resection of rib osteochondroma, and postoperative complications such as intercostal neuralgia did not occur. In 2019, Tsakotos et al. [28] reported two cases of extra-articular osteochondroma of the distal femur, which was removed by arthroscopic surgery, but they entered the joint through a conventional knee arthroscopic approach first, and then, a hole was punched on the joint capsule to pass through the vastus medialis muscle to the mass site. However, we found that most of the reports on arthroscopic resection of extra-articular osteochondroma are case reports, and there are few comparatively systematic follow-up and analysis studies, let alone multi-dimensional functional evaluation on patients. The author’s department focuses on sports medicine clinical and scientific research and has tried the application of arthroscopy in extra-articular osteochondroma for years [10,29]. Our surgical approach is to create two arthroscopic portals with an interval of 3 cm directly on the surface of the tumor, without entering the joint, avoiding damaging important structures. Among the 74 patients, the postoperative VAS score was significantly lower than that before operation (*p* < 0.001); the Lysholm score, IKDC score, and Tegner score were significantly improved compared with those before operation, with no tumor recurrence or metastasis occurred in all patients during the follow-up.

In order to achieve better surgical results, there are many tips to which attention should be paid. Firstly, the preoperative preparation and evaluation of arthroscopic resection of benign bone tumors are very important, and the indications and contraindications of the operation should be strictly controlled. The most important point is that the nature of the tumor must be determined before surgery. For the common bone tumors, the nature of the tumor can often be determined by imageological examinations, such as osteochondroma, giant cell tumor of bone, etc. [30]. However, for tumors with atypical clinical manifestations for which the nature cannot be confirmed by imageological examination, pathology is required before surgery, and arthroscopic treatment can only be performed after it is clear that the bone tumor is benign [31]. Secondly, it is necessary to accurately locate the tumor and measure the size of the tumor before the operation so as to facilitate the location of the incision and the preoperative selection of appropriate tools for tumor resection under the microscope. Furthermore, it is necessary to use MRI or ultrasound to determine whether there are major blood vessels or nerves in the vicinity of the tumor before surgery so as to determine whether it is suitable for arthroscopic surgery as well as the position and operation direction of the incision to avoid blood vessels and nerves damage [32].

Besides preoperative evaluation, intraoperative re-evaluation of the tumor is also very important. If there is a significant difference between the intraoperative findings and the preoperative judgment, it must decisively change to open surgery or other surgical methods. In addition, during the whole operation, it is necessary to maintain sufficient and smooth drainage of the perfusate to minimize the infiltration and spread of perfusate to surrounding tissues so as to avoid tumors’ spreading and metastasis [17].

We all know that the important structure for the growth of osteochondroma and postoperative recurrence is the cartilage cap, so the key procedure is to completely remove the cartilage cap to prevent its recurrence [33]. Therefore, for this technique, our experience is that the cartilage cap should be completely burned with a radiofrequency knife after the tumor is fully exposed. For the rest of the tumor, one may choose to chisel from the root or gradually cut with nucleus forceps pulposus and finally remove a little normal bone at the root edge of the tumor to further ensure that it will not relapse.

In conclusion, we believe that arthroscopic resection of osteochondroma is less traumatic because it can accurately and completely remove tumors. It is a new, safe, and feasible surgical method to remove osteochondroma with only a small local scar, quick functional recovery, mild pain, and no recurrence or metastasis for not only for osteochondromas but also for most of the benign bone tumors. In addition to its minimally invasive nature, arthroscopic resection of benign bone tumors also has high definition, and surgeons can clearly distinguish the boundary between the tumor and normal tissue; moreover, this technique can clearly show whether the tumor has been completely removed. However, it should be noted that the surgical indications must be strictly controlled. For osteochondromas or other benign bone tumors that are prone to recurrence, tend to be malignant, or are adjacent to important blood vessels and nerves, it is recommended to use open surgery instead. The pursuit of less invasive techniques must not lead to greater trauma.

## Figures and Tables

**Figure 1:** Image data of arthroscopic resection of extra-articular osteochondroma of the knee. (**A**) Preoperative X-ray can clearly show osteochondroma, and the tumor and surrounding tissue are clearly demarcated; (**B**) the tumor can be clearly observed by arthroscopy during the operation. (**C**) A small tumor was removed with rongeur. The tissue was sent to rapid pathological examination during the operation. (**D**) The tumor tissue was gradually removed with rongeur, and a few normal bones were removed. (**E**) The tumor tissue was completely removed to reduce the cell spreading. (**F**) Two small incisions. (**G**) Postoperative review of X-ray showed that the tumor had been completely removed. (**H**) Osteochondroma was confirmed after postoperative pathological examination.

**Table 1:** Knee pain and function scores at each follow-up time point.

	Preoperative	3 Months after Surgery	6 Months after Surgery	12 Months after Surgery	≥24 Months after Surgery	*p*-Value
VAS	3.6 ± 1.1	1.3 ± 0.6 *	0.5 ± 0.1 *^/^**	0.3 ± 0.06 *^/^**	0.1 ± 0.02 *^/^**	<0.001
Lysholm	44.5 ± 2.3	70.1 ± 3.6 *	87.9 ± 4.2 *^/^**	90.2 ± 4.7 *^/^**	91.3 ± 4.9 *^/^**	<0.001
IKDC	53.7 ± 2.6	82.1 ± 3.7 *	88.9 ± 4.1 *^/^**	92.4 ± 4.6 *^/^**	94.2 ± 5.1 *^/^**	<0.001
Tegner	4.6 ± 1.2	6.5 ± 1.4 *	8.0 ± 1.6 *	8.9 ± 2.0 *^/^**	9.4 ± 1.4 *^/^**	<0.001

Note: * Compared with preoperative, the difference is statistically significant; ** compared with 3 months after operation, the difference is statistically significant. IKDC: International Knee Documentation Committee. VAS: visual analog scale.

## Data Availability

The data associated with the paper are not publicly available but are available from the corresponding author upon reasonable request.
